RETRACTED

# Predictability of combined cataract surgery and trabeculectomy using Barrett Universal Ⅱ formula

**DOI:** 10.1371/journal.pone.0270363

**Published:** 2022-06-23

**Authors:** Kei Iijima, Kazutaka Kamiya, Yoshihiko Iida, Masayuki Kasahara, Nobuyuki Shoji

**Affiliations:** 1 Department of Ophthalmology, Kitasato University, Sagamihara, Japan; 2 Visual Physiology, School of Allied Health Sciences, Kitasato University, Sagamihara, Japan; Cairo University Kasr Alainy Faculty of Medicine, EGYPT

## Abstract

**Purpose:**

To compare the predictability of intraocular lens (IOL) power calculation using the Barrett Universal II and the SRK/T formulas in eyes undergoing combined cataract surgery and trabeculectomy.

**Methods:**

We retrospectively reviewed the clinical charts of 56 consecutive eyes undergoing cataract surgery and trabeculectomy. IOL power calculations were performed using the Barrett Universal II and SRK/T formulas. We compared the prediction error, the absolute error, and the percentages within ± 0.5 D and ±1.0 D of the targeted refraction, 3 months postoperatively, and also investigated the relationship of the prediction error with the keratometric readings and axial length, using the two formulas.

**Results:**

The prediction error using the SRK/T formula was significantly more myopic than that using the Barrett Universal II formula (paired t-test, p<0.001). The absolute error using the Barrett Universal II formula was significantly smaller than that using the SRK/T formula (p = 0.039). We found significant correlations of the prediction error with the axial length (Pearson correlation coefficient, r = 0.273, p = 0.042), and the keratometric readings (r = -0.317, p = 0.017), using SRK/T formula, but no significant correlations between them (r = 0.219, p = 0.167, and r = -0.023, p = 0.870), using the Barrett Universal II formula.

**Conclusions:**

The Barrett Universal II formula provides a better predictability of IOL power calculation and is less susceptible to the effect of the axial length and the corneal shape, than the SRK/T formula. The Barrett Universal formula, rather than the SRK/T formula, may be clinically helpful for improving the refractive accuracy in such eyes.

## Introduction

Cataract surgery has become a widely recognized refractive surgery, since the safety and the efficacy has been much improved, and subsequent patient expectation has become higher year by year. In order to correct refractive errors as much as possible, it is mandatory to accurately calculate the IOL power using modern sophisticated calculation formulas. In recent years, the Barrett Universal II formula has been gathering attention to provide more accurate IOL power than other conventional formulas [1–4].

RETRACTED

To date, there have been only a few studies on the predictability of combined cataract surgery and trabeculectomy, but all these studies merely focused on the refractive error by using conventional IOL power calculation formulas, such as the SRK II, SRK/T Holladay, and Hoffer Q formulas [5–7]. However, to the best of our knowledge, the Barrett Universal II formula has not been applied for these combined surgical procedures. It may give us intrinsic insights on the IOL power calculation of modern cataract surgery with trabeculectomy, which is one of the viable surgical options in eyes having coexisting cataract and glaucoma.

In the present study, our goal is twofold; to assess the predictability outcomes of combined cataract surgery and trabeculectomy using the Barrett Universal II formula, with special attention to the keratometric readings and axial length, and to compare the outcomes with them using the SRK/T formula.

## Materials and methods

### Study population

The study protocol was registered with the University Hospital Medical Information Network Clinical Trial Registry (000038822). This retrospective study comprised a total of 56 eyes of 56 consecutive patients (24 men and 32 women, mean age ± standard deviation: 69.1 ± 7.8 years), who underwent simultaneous cataract surgery and trabeculectomy with non-toric monofocal IOL implantation, between June 2015 and June 2019 at Kitasato University Hospital, and who completed a 3-month follow-up. Eyes with postoperative best corrected visual acuity of >0.15 logMAR, eyes with any history of ocular surgery, ocular trauma, or other concomitant eye diseases, and eyes developing any intraoperative or postoperative complications that could affect refractive outcomes, were excluded from the study. This retrospective review of the data was approved by the Institutional Review Board at Kitasato University (B19-200) and followed the tenets of the Declaration of Helsinki. Our Institutional Review Board waived the requirement for informed consent for this retrospective study.

### Surgical procedures

Experienced surgeons conducted standard phacoemulsification, followed by IOL power calculation. The surgical technique consisted of a capsulorhexis, nucleus and cortex extraction, and non-toric IOL (AQ-110NV, STAAR Surgical, Chiba, Japan) implantation, through a 2.8-mm temporal corneal incision. One 11–0 nylon suture was placed to prevent leakage from corneal incision.

Simultaneously, they conducted standard trabeculectomy with a nasal superior fornix-based conjunctival flap and partial thickness rectangular scleral flap (3.0 x 3.0 mm). In all cases, 0.5 mg/mL of mitomycin-C was applied for 2 minutes. The scleral flap and conjunctiva were sutured with 4 to 6 interrupted 10–0 nylon sutures. Postoperative suture lysis was appropriately performed to achieve that the intraocular pressure was maintained between 10 and 12 mmHg. Postoperatively, steroidal, antibiotic, and bromfenac sodium medications were topically administered for 1 month, the dose being reduced gradually thereafter.

RETRACTED

### Assessment of prediction error and absolute error

We performed IOL power calculations by using the Barrett universal Ⅱ formula and SRK/T formula, using axial length, keratometric readings (for both formulas), and anterior chamber depth (only for Barrett Universal II formula), measured with a partial coherence interferometer (IOL Master 500^TM^, Carl Zeiss Meditec, Jena, Germany). We used the optimized A-constants for the IOL power calculation. The prediction errors defined by subtracting the predicted postoperative refraction from the postoperative spherical equivalent 3 months postoperatively, these absolute values, and the percentages of eyes within ± 0.5 D and ±1.0 D of the targeted refraction, were calculated [8, 9].

We also assessed the relationship between the prediction error and the keratometric readings and axial length, in order to clarify the effect of the keratometry or axial length on the refractive accuracy, using the two IOL formulas.

### Statistical analysis

We performed statistical analyses by using a commercially available statistical software (Bellcurve for Excel, Social Survey Research Information Co, Ltd., Tokyo, Japan). Since normal distribution of the data was confirmed by the Kolmogorov-Smirnov test, the paired t-test was used to compare the prediction errors using the two IOL power calculation formulas. The Pearson correlation coefficient was used to assess the relationship of the two variables. The Fisher’s exact test was used to compare the percentages of eyes within ± 0.5 D and ±1.0 D of the targeted correction. The results are expressed as mean ± standard deviation, and a value of p<0.05 was considered statistically significant.

## Results

Table 1 shows the preoperative demographics of the study population. The intraocular pressure was significantly decreased, from 17.8 ± 4.7 mmHg preoperatively, to 11.0 ± 3.0 mmHg postoperatively (paired t-test, p<0.001). The prediction error (-0.35 ± 0.65 D) using the SRK/T formula was significantly more myopic than that (-0.09 ± 0.34 D) using the Barrett Universal II formula (p<0.001) (Fig 1). The absolute error (0.46 ± 0.13 D) using the Barrett Universal II formula was significantly smaller than that (0.56 ± 0.47 D) using the SRK/T formula (p = 0.039) (Fig 2). The percentages within ± 0.5 D and ± 1.0 D of the targeted refraction were 54 and 79%, respectively, using the SRK/T formula, and 63% and 91%, respectively, using the Barrett Universal II formula. There were no significant differences in the percentages within ± 0.5 D and ± 1.0 D using the two formulas (Fisher’s exact test, p = 0.444, p = 0.127).

RETRACTED

**Fig 1:** A graph showing the prediction error using the SRK/T and the Barrett Universal II formulas. The prediction error using the Barrett Universal II formula was significantly more myopic than that using the SRK/T formula (paired t-test, p<0.001).

**Fig 2:** A graph showing the absolute error using the SRK/T and the Barrett Universal II formulas. The absolute error using the Barrett Universal II formula was significantly smaller than that using the SRK/T formula (paired t-test, p = 0.022).

**Table 1:** The preoperative demographics of the study population.

Mean ± standard deviation (range)	
Number of eyes	56
Age	69.1 ± 7.8 years (51 to 82 years)
Male: Female	24: 32
logMAR CDVA	0.07 ± 0.12 (-0.08 to 0.40)
Mean keratometric readings	44.65 ± 1.39 D (41.33 to 48.23 D)
Axial length	24.81 ± 1.78 mm (21.37 to 28.93 mm)
Intraocular pressure	17.8 ± 4.7 mmHg (11 to 35 mmHg)
Glaucoma type (POAG: NTG: CACG: PESG)	33: 16: 3: 4

logMAR = logarithm of the minimal angle of resolution, CDVA = corrected distance visual acuity, D = diopter, POAG = primary open angle glaucoma, NTG = normal tension glaucoma, CACG = chronic angle closure glaucoma, PESG = pseudo-exfoliation secondary glaucoma.

We found a significant positive correlation between the prediction error and the axial length using the SRK/T formula (Pearson correlation coefficient, r = 0.273, p = 0.042), but no significant correlation between them using the Barrett Universal II formula (r = 0.219, p = 0.167) (Fig 3). We also found a significant negative correlation between the prediction error and the keratometric readings using the SRK/T formula (r = -0.317, p = 0.017), but no significant correlation between them using the Barrett Universal II formula (r = -0.023, p = 0.870) (Fig 4).

**Fig 3:** A graph showing correlations between the prediction error and the axial length (Pearson correlation coefficient, r = 0.219, p = 0.167 for the Barrett Universal II formula, r = 0.273, p = 0.042 for the SRK/T formula).

**Fig 4:** A graph showing correlations between the prediction error and the mean keratometry (Pearson correlation coefficient, r = -0.023, p = 0.870 for the Barrett Universal II formula, r = -0.317, p = 0.017 for the SRK/T formula).

## Discussion

In the present study, our results showed that the use of the Barrett Universal Ⅱ formula provided a higher predictability of IOL power calculation than that of the SRK/T formula, in terms of the prediction and absolute errors. Our results also showed that there were significant correlations of the prediction error with the axial length and the keratometric readings using the SRK/T formula, but no significant correlations between them using the Barrett Universal II formula. It is suggested that the SRK/T formula was susceptible to the axial length and the keratometric readings, but the Barrett Universal II formula was not susceptible to them, even in eyes undergoing combined cataract surgery and trabeculectomy. It was in agreement with previous studies on cataract surgery alone. Olsen et al. [10] demonstrated that the SRK/T formula showed a hyperopic error in eyes with long axial length (>26.0 mm). Zhang et al. [11] showed that Barrett Universal II formula provided the lowest predictive error and the least variable predictive error compared with the SRK/T and other formulas in high myopic eyes. Liu et al. [12] showed that the percentage of eyes (79.56%) within 0.5 D using the Barrett Universal II formula was significantly higher than that (61.88%) using the SRK/T formula in eyes with long axial length (>26.0 mm). Olsen et al. [10] found a significant negative correlation of the prediction error with the keratometric readings (r = -0.23, p<0.0001), when the SRK/T formula was used. Faramarzi et al. [13] demonstrated that the prediction error was -0.06 ± 0.52 D in eyes with a keratometry > 46 D, when the SRK/T formula was applied. Reitblat et al. [14] showed that myopic refractive errors (-0.31 ± 0.54 D) were found in eyes with a keratometry > 46 D, but hyperopic errors (0.16 ± 0.31 D) were observed in eyes with a keratometry < 42 D, when the SRK/T formula was used, and that the prediction error was -0.04 ± 0.45 D and -0.07 ± 0.26 D, in eyes with a keratometry > 46 D and < 42 D, respectively, both of which were not significantly different from zero, when the Barrett Universal II formula was used.

RETRACTED

Table 2 summarizes previous studies on the predictability of simultaneous cataract surgery and trabeculectomy [5–7]. Law et al. [5] demonstrated that the refractive outcome of combined cataract surgery and trabeculectomy did not differ significantly from the predicted refraction in comparison with cataract surgery alone, using the average IOL power obtained from the results of the SRK/T, Holladay, and Hoffer Q formulas. Chan et al. [6] showed that the prediction and absolute errors after phacotrabeculectomy were 0.20 ± 1.31 D and 0.96 ± 0.89 D, respectively, using the SRK II formula. Chung et al. [7] stated that the prediction and absolute errors after phacotrabeculectomy were -0.05 ± 0.64 D and 0.46 ± 0.44 D, respectively, using the SRK/T formula. However, conventional IOL power calculation formulas were used in all previous studies. As far as we can ascertain, this is the first report to assess the refractive accuracy of combined cataract surgery and trabeculectomy using the latest Barrett Universal II formula, which has been reported to provide higher accuracy of IOL power calculation than conventional formulas. Moreover, we only included eyes with postoperative logMAR CDVA ≤ 0.15 in this study, since accurate and reliable refraction could be obtained. In consideration of the strict inclusion criteria, we believe that it will be helpful for improving the predictability of these combined procedures in daily practice.

**Table 2:** Summary of previous studies on the predictability of intraocular lens power calculation in eyes undergoing combined cataract surgery and trabeculectomy.

Author	Number of eyes	IOL power calculation formula	Inclusion criteria (Postoperative logMAR CDVA)	Prediction error (D)	Within ± 0.5 D (%)	Within ± 1.0 D (%)
Law SK et al. [5]	24	SRK/T, Holladay, and Hoffer Q	N.A.	0.22 ± 0.91	N.A.	N.A.
Chan JC et al. [6]	25	SRK II	N.A.	0.20 ± 1.31	N.A.	N.A.
Chung JK et al. [7]	51	SRK/T	< 1.00	-0.05 ± 0.64	67	90
Current	56	Barrett Universal II	≤ 0.15	-0.09 ± 0.34	63	91
		SRK/T		-0.35 ± 0.65	54	79

IOL = intraocular lens, logMAR = logarithm of the minimal angle of resolution, CDVA = corrected distance visual acuity, D = diopter, N.A. = not applicable.

There are several limitations to this study. First, the study was performed in a retrospective fashion. Second, the sample size was relatively small. A prospective study with a large number of patients would be helpful for confirming the authenticity of our results. Third, we did not investigate the effect of the changes in keratometry or axial length on the predictability outcomes, since we primarily focused on the refractive outcomes of combined cataract surgery and trabeculectomy. Fourth, we did not have a control group of cataract surgery alone. Therefore, the effect of trabeculectomy itself on the refractive accuracy remained unanswered. Fifth, we did not use the intraoperative abberometry for IOL power calculation. It has been reported that the mean absolute error using the intraoperative aberrometry was significantly lower than that using the preoperative biometry in a total of 32189 eyes [15]. Therefore, it would be beneficial for further improving the predictability in eyes undergoing such combined surgical procedures.

In conclusion, our results may support the view that the Barrett Universal II formula provides a higher predictability of the IOL power calculation than the SRK/T formula, and that the former formula is less susceptible to the axial length and the keratometric readings than the latter formula, even in eyes undergoing combined cataract surgery and trabeculectomy. We believe that this information may be clinically helpful for understanding the properties of the two major IOL power calculation formulas in eyes requiring combined cataract surgery and trabeculectomy.
